# The nexus of environmental sustainability and agro-economic performance of Sub-Saharan African countries

**DOI:** 10.1016/j.heliyon.2020.e04878

**Published:** 2020-09-14

**Authors:** Festus Fatai Adedoyin, Andrew Adewale Alola, Festus Victor Bekun

**Affiliations:** a Department of Accounting, Economics and Finance, Bournemouth University, United Kingdom; b Faculty of Economics Administrative and Social Sciences, Istanbul Gelisim University, Istanbul, Turkey; c Department of Financial Technologies, South Ural State University, Chelyabinsk, Russia; d Department of Accounting, Analysis and Audit, School of Economics and Management, South Ural State University, 76, Lenin Aven., Chelyabinsk 454080, Russia

**Keywords:** Environmental science, Economics, Agricultural value added, Urbanization, Total natural rent, Carbon emissions, Sub-Saharan African countries

## Abstract

The increasing concern of environmental degradation and climate change impacts of agricultural-based activities are becoming more pronounced in the Sub-Sahara region of Africa especially due to urgent drive to meeting food, healthy diet, and economic needs. In retrospect. This novel study explores the relationship between agro-economic performance, the Real Gross Domestic Product (GDP), Total natural rent, urbanization and environmental degradation vis-à-vis (Carbon dioxide emissions) in a carbon function. The empirical analysis used a panel data for the period 1980–2014 for the selected countries in sub-Saharan Africa. The Kao test uncovers a cointegration between carbon dioxide emissions, Real Gross domestic product, Total natural rent, agriculture and urbanization. The panel Pooled Mean Autoregressive distributed lag model (PMG-ARDL) posits a positive and significant connection between the gross domestic product and CO_2_ emissions in the long run. Our examination asserts that agricultural value-added reduces emissions in sub-Saharan Africa while urbanization and natural resource rent both increases CO_2_ emissions in the long run. In addition, the causality analysis reveals a bidirectional link between agriculture value-added and CO_2_ emissions. Essentially, policymakers in African nations must pay close attention to the issues of rural-urban drift as this leads to more emissions.

## 1 Introduction

The grave implications of climate change to humans and the ecosystems has remained a source of concern to research scholars, as well as generating public debates. The greenhouse effect is considered the lead contributor to global warming because it is a natural process that significantly increases the temperature of the earth surface through the accumulation of atmospheric heat (Apergis and Payne, 2009; Ozturk, 2010; Kweku et al., 2018; Alola, 2019a, Alola, 2019b; Alola et al., 2019a, Alola et al., 2019b). This has continued especially with incessant rise in agricultural mechanization (Olasehinde-Williams et al., 2020). Carbon dioxide (CO_2_), Methane, Fluorinated gases and Nitrous Oxide are some of the gases that majorly contributes to the greenhouse effect. A report by the U.S Environmental Protection Agency (2019) also shows that Carbon dioxide contributes about 82% of the overall greenhouse emissions in 2017 as shown in Figure 1 below (United States Environmental Protection Agency (EPA), 2017). This shows that a major causative agent of climate change is carbon dioxide emission. Moreover, Tutmez (2006) stated that, though carbon dioxide accounts for about 0.03 per cent of the earth's atmospheric volume, its percentage has increased by 25 per cent even before the industrial age. The rapid increase in population, energy demand, economic growth, and agricultural production over the decades is largely responsible for the significant increase in carbon dioxide emissions in the atmosphere (Appiah et al., 2018). This implies that the amount of heat trapped in the atmosphere is in the upward trend. In the case of Sub-Saharan Africa, for instance, Demissew Beyene and Kotosz (2019) noted that carbon dioxide emissions have reached their peak between the year 1990 and 2014 (precisely in 2003). However, the study expressed that a decline in carbon emissions was experienced in Sub-Saharan Africa between 2007 and 2013 before starting to increase again in the year 2014.

**Figure 1:** United States Environmental Protection Agency (EPA), 2017: Overview of greenhouse gas emissions in 2017 (%).

Considering that the International Monetary Fund (IMF) (2012) opined that more than half of the labour force in Sub Saharan Africa is employed in the agricultural sector (accounting for more than 60 per cent), this highlights the importance of the sector to the region's economy. Agricultural sector's share in the Gross Domestic Product for Sub Saharan Africa in 2009 was 12.7 per cent. This suggests the reason most of the continent's economic drive at achieving sustainable development growth is significantly hinged on the agricultural sector. Moreover, the World Bank (2019) opined that 80 per cent of the world's poor, who lives in rural communities can reduce poverty, food insecurity, and raise their income through agriculture. Interestingly, in 2017, Africa's economy recorded an average growth rebound to 3.4 per cent (a 0.9 per cent increase in growth rate) with an expected estimate of 4.3 per cent in 2018. Thus, this positioned Africa in second place among the fastest-growing economy in the world (Africa Development Bank, AfDB, 2017). However, with the importance of the agricultural sector to the development of Africa, the continent is still generally lagging in its productivity due to challenges associated with the continent's agricultural system.

On the other hand, the spate of population growth in Africa has remained a source of concern. On the account of Jerusalem (2016), the population of the Sub Saharan Africa in 2050 would almost be 2.1 billion in contrast to its figure in 2016, which is 950 million. Unfortunately, this increase is not without its burdens. For instance, the explosion in human population over the years has resulted in a high rate of urbanization. The urban cities are expanding, thereby occupying sizable lands that could be used for agricultural purposes Olasehinde-Williams et al. (2020). This effect has deprived farmers of the liberality of practicing shifting cultivation. Thus, the excessive use of specified arable land over a long period reportedly contribute immensely to environmental pollution due to the release of pollutant gases that affects the atmosphere. Also, the issue of undernourishment in Sub Saharan Africa has a very long history. In 2016, an estimate of undernourished persons was reported as 218 million with an increase of 44 million (Jerusalem, 2016). Therefore, to meet the demand of feeding the population and solve the problem of undernourishment, agricultural activities and productivities are expected to increase drastically. Furthermore, urbanization could be associated with diversity in the pattern of food consumption in the city. There is an increase in the consumption of processed foods, convenience foods, fast foods and so on (FAO-ONU, 2017). Another effect of urbanization is deforestation. Tropical deforestation contributes about 20 per cent of the greenhouse emissions (Derouin, 2019). These among other reasons signalled the renewed agreement of the United Nations Framework Convention on Climate Change (UNFCCC) in March 2019 that aids further commitment to keeping the rise in global mean temperature level below 2 °C. Other parts of the commitment include increasing renewable energy consumption shares by 20 per cent, and increasing energy efficiency thereby saving up to 20 per cent of energy consumption (Ozturk, 2010; Asongu et al., 2016; Asongu et al., 2017; Alola and Alola, 2018; Agboola and Bekun, 2019, Alola, Yalçiner & Alola, 2019).

To drive down the above motivation, the current study is aimed at testing the effect of agricultural activates and the economic performance of the Sub-Sahara Africa countries as a way of enhancing policies that will help in recovering our blue skies. As a mark of novelty, the study is foremost in examining the potential effect of agricultural-based activities on environmental quality for the very important case of Sub-Sahara. Additionally, the novelty of the study is fine-tuned by further examining the evidence of the Environmental Kuznets Curve (EKC) hypothesis for the Sub-Sahara region of Africa. Moreover, this investigation was carried out not without looking at the impact of urbanization and total resource rent on environmental quality in the region. As such, the contribution of this study is that it attempts to uncover key procedures that countries in Sub-Saharan Africa can embrace toward accomplishing rural sustainable development and simultaneously moderate the adverse impact of agricultural activities for the earth.

The remainder of the study involves the theoretical underpinning of agriculture-induced pollutant emissions in section two. In section three and four, the empirical models, methods and data description are presented while the discussion of results is outlined in section five. A concluding remark with policy recommendations is presented in section five.

## 2 Theoretical perspective

The theoretical theme for this study revolves around the Environmental Kuznets curve Hypothesis. The environmental Kuznets (EKC) hypothesis entails the inverse relationship between per capita income level and environmental quality. It explains the inverse impact of the economic growth trajectory on the environment. Discovered by Kuznets (1955) the hypothesis is observed in three paths: the scale effect, composite effect and technique effect. The first stage which is the scale effect entails the initial developmental period in an economy whereby there is much emphasis on economic expansion relative to environmental quality (Azam and Khan, 2016; Shahbaz & Sinha, 2019). This stage is more related to developing countries where the awareness of the need to maintain the quality of the environment is minimal, while the majority of the economic activities are in the primary sector; mining, agricultural activities which in constitute a huge source of pollution to the environment.

The second stage known as the composite stage encompasses a higher level of industrial activities and economic development whereby some level of consciousness concerning the environment is maintained. Emerging economies fall within this tier. The third phase is the technique scale where countries begin to observe a reduction in environmental pollution as they reach a ‘turning point threshold’ (Shahbaz & Sinha, 2019). At this stage, countries begin to adopt cleaner energy as well as begin to regulate economic activities in a way that will continue to improve the quality of the environment. Developed countries have made it to this stage.

Several variables have been included in the EKC model such as agricultural output (Kaczan et al., 2013; Kim et al., 2015; Asumadu-Sarkodie and Owusu, 2016; Bennetzen et al., 2016; Li et al., 2016; Mehdi and Slim, 2017; Gokmenoglu and Taspinar, 2018; Agboola and Bekun, 2019; Ben Jebli et al., 2020), urbanization (Wang et al., 2019) and natural resource rent (Bekun et al., 2019; Balsalobre-Lorente et al., 2018). The role of agriculture in the EKC is explained through its relationship with economic growth. As explained by Adebola and Bekun, (2019). Agriculture is an economic activity which processes involve the emission of greenhouse gases into the atmosphere. Hence, agricultural value-added is expected to have a positive impact on emissions. The role of Urbanization on emissions is explained via the urban environmental transition theory where the expansion of cities leads to an expansion in manufacturing activities; leading to massive air and water pollution (Abdallh and Abugamos, 2017). Few studies found a negative impact of urbanization on emissions. While a study by Wang et al. (2019) found a positive relationship between urbanization and emissions.

The role of natural resources on environmental pollution is traced through its impact on economic growth in a country (Sachs and Warner, 1995; 1997; Sala-i-Martin et al., 2004). As such some attempts have been made to include the role of natural resources in the EKC leading to various conclusions (Bekun et al., 2019; Balsalobre-Lorente et al., 2018). While the study of Bekun et al. (2019) finds that natural resources aggravates the level of emissions in the environment, that of Balsalobre-Lorente et al. (2018) argues that natural resource rents lead to an improvement in the environment. While several studies have shown emissions arising from several factors (F. Adedoyin et al., 2020b, 2020a; Adedoyin et al., 2020c, 2020d, 2020e; Adedoyin and Zakari, 2020; Etokakpan et al., 2020; Kirikkaleli et al., 2020; Udi et al., 2020), there are two ways to control carbon dioxide and other greenhouse gas emissions from energy usage in agriculture (Li et al., 2016), one is to increase the efficiency of the energy, the other is to increase renewable energy usage.

## 3 Data and methodology

### 3.1 Data

Our investigation utilizes panel data that is balanced for the combination of 12 sub-Saharan African countries over the period under consideration 1980–2014. The estimation model uses carbon dioxide outflows (CO_2_) as the dependent variable. The independent variables utilized are Real Gross domestic product; Agricultural value-added; Urbanization; Total natural rent. In the estimation model, the unobserved components are controlled for by real Gross domestic product per capita. The World Bank (2017) Development indicator is the source of the data series. Information accessibility (particularly for emissions) is to a great extent answerable for both the limited time of the data arrangement and the choice of the assessed nations which include Benin; Cote d'ivoire; Mauritius; Botswana; Ethiopia; Nigeria; Cameroon; Ghana; South Africa; Congo Republic; Kenya and Zimbabwe. See Table 1 for an outline of the description of variables used.

**Table 1:** Indicators and unit of measurement.

Variables	Code	unit of measurement	Source
Real Gross domestic product	GDP	constant 2010 $ USD	WDI
Agricultural value added	AG	% of total final energy	WDI
Urbanization	URB	(% of total)	WDI
Total natural rent	NRT	(%GDP)	WDI
Carbon dioxide emissions	CO_2_	(Kt)	WDI

Note: WDI represents world development indicator (https://data.worldbank.org/).

### 3.2 Estimation process

The test process utilized is structured as follows:(i) We tested for stationarity among the interest variables using the Fisher-ADF, Levin, Lin and Chu (LLC) and the Im et al. (2003) unit root tests. This is to avoid a spurious regression arising from the presence of I (2) stationary variables. (ii) We examined for the existence of a long-run equilibrium relationship among the variables in the model by using the Pedroni cointegration test by Pedroni (1999) and the Kao cointegration for robustness. (iii) Given the existence of cointegrating relationships from the results obtained in (iv), we estimated long and short-run equilibrium relationship via the panel pooled mean group estimator by Pesaran et al. (1999) and (iv) we investigated the direction of causation among the variables through the Dumitrescu and Hurlin (2012) causality test. Before the unit root tests, the study performed the summary statistics for the variables to reveal the characteristics of the series. Also, the variables were subjected to the Pearson correlation matrix analysis to examine the linear association among the variables.

### 3.3 Model estimation

While several studies have assessed the nexus of emissions-growth and energy consumption (Adedoyin et al., 2020e, 2020a), the current study introduces agriculture induced emissions with a special focus on selected countries in sub-Saharan Africa using a large span of data. Furthermore, our model remarkably consolidated resource rent and agriculture value-added and urbanization in the investigation with the end goal that:

(1) $$LCO2_{it}=\beta_{0}+\beta_{1}LGDP_{it}+\beta_{2}LGDP2_{it}+\beta_{3}LAGR_{it}+\beta_{4}LURB_{it}+\beta_{5}LNRT_{it}+\varepsilon_{it}$$

For the data to have a consistent variance, the investigation applies a logarithmic change. Here, LCO_2_, LGDP, LGDP2, LAGR, LURB, and LNRT indicate the logarithmic transformation of the variables, $\beta_{0}$ relates to the constant term, while β′s 1 to 5 are the slope coefficients, and ε_it_ is the stochastic term. Because of bias activated by the connection between the mean-differenced autonomous factors and the disturbance term, standard ARDL estimation models are unequipped for controlling for such bias particularly in panel data models with singular impacts. In that capacity, the PMG estimator by Pesaran et al. (1999) is therefore employed for its uniqueness to model series with integrated order at the level and first difference or a mixture of both orders. Additionally, the ARDL/PMG estimator is robust as it simultaneously presents a long and short-run dynamic analysis. Finally, the ARDL-PMG approach is also reportedly suitable for short sample analysis. Despite existing panel data models accessible in (Azam, 2019; Destek and Sarkodie, 2019; Bekun et al., 2019), this examination follows the PMG-ARDL pathway used in (Sarkodie and Strezov, 2018), communicated as:

(2) $$\text{Δ}lny_{it}=\emptyset_{i}ECT_{it}+\sum_{j=0}^{q-1}\text{Δ}lnX_{1\left(t-j\right)}\beta_{ij}+\sum_{j=1}^{p-1}\psi_{ij}\text{Δ}lny_{i\left(t-j\right)}+\varepsilon_{it}$$

(3) $$ECT_{it}=y_{i\left(t-1\right)}-X_{it}\theta$$

where y is the regressed variable (LCO2), X relates to the regressors (Gross domestic product, Agriculture value-added, resource rent and urbanization) with the same number of slacks q across singular cross-sectional units *i* in time *t*, Δ denotes the difference operator, φ is the alteration or adjustment coefficient, θ indicates the long term coefficient that produces β and ψ appraises the behaviour of the model after reaching convergence while ε is the error term. This examination follows 3 ways for its empirical investigation. (I) Stationarity test by fisher ADF and Pesaran et al. (2003) unit root test (ii) cointegration examination and long-run analysis progressed by Pesaran et al. (1999) and (iii) Causality investigation through Dumitrescu and Hurlin (2012). In any case, a primer estimation of summary statistics and correlation matrix were carried out.

## 4 Results and discussions

### 4.1 Preliminary results

The quality of the dataset used for the empirical analysis is investigated, and the descriptive statistics of each of the variables, namely carbon dioxide emissions (CO_2_), real gross domestic product (GDP), agricultural value-added (AG), urbanization (URB), and total natural rent (NRT) are presented in Table 2. The average value of carbon dioxide emission in sub-Saharan African countries stands at 41483.48. This value is very high compared to the mean values of real gross domestic product (7343.99), agricultural value-added (20.66), urbanization (38.71), and total natural rent (11.695). Additionally, carbon dioxide emission has the highest minimum value (407.04), while total natural rent has a minimum (0.001). It can also be observed from the result that carbon dioxide emission has the highest maximum values (503112.40) followed by real gross domestic product (2142693.00). This is a reflection of the environmental degradation in sub-Saharan African countries. Further, the values of the skewness suggest that the distribution of each of the variables is skewed to the right except urbanization that has a negative coefficient. Also, the result shows that all the variables have the same number of observations.

**Table 2:** Summary Statistics and Correlation analysis.

	CO_2_	GDP	AG	URB	NRT
Mean	41483.480	7343.989	20.662	38.711	11.695
Median	5210.807	1309.064	20.659	40.680	7.133
Maximum	503112.400	2142693.000	63.831	66.368	63.550
Minimum	407.037	163.623	1.828	10.410	0.001
Std. Dev.	105065.300	104463.400	14.250	13.821	12.961
Skewness	3.059	20.409	0.664	-0.197	1.888
Kurtosis	11.160	417.677	2.835	2.283	6.086
Jarque-Bera	1820.382	3038405.000	31.359	11.696	416.102
Probability	0.000	0.000	0.000	0.003	0.000
Observations	420	420	420	420	420

Correlation coefficient analysis					

CO_2_	1				
GDP	-0.007	1.000			
AG	-0.347	0.102	1.000		
URB	0.362	-0.088	-0.662	1.000	
NRT	-0.073	-0.003	0.015	0.139	1

Table 2 also reports the coefficients of the correlation matrix for carbon dioxide emissions, real gross domestic product, agricultural value-added, urbanization, and total natural rent. The result of the analysis indicates that real gross domestic product, agricultural value-added, and total natural rent are negatively correlated with carbon dioxide emission. At the same time, urbanization has a positive association with carbon dioxide emissions in sub-Saharan African countries. Further, agricultural value-added and urbanization are found to be strongly correlated with carbon dioxide emissions compared to real gross domestic product and total natural rent. The strong negative relationship between agricultural value-added and carbon dioxide proves that a clean environment can be achieved with agrarian in sub-Saharan African countries.

#### 4.1.1 Unit root test

The stationary test is a prerequisite for panel data analysis. So, to ascertain the order at which carbon dioxide emissions, real gross domestic product, agricultural value-added, urbanization, and total natural rent are stationary, the study employs three-panel unit root tests. These tests are Fisher-ADF, Levin, Lin and Chu (LLC) and Im, Pesaran and Shin (IPS). Table 3 reports the results of the tests for the level and first difference stationary (constant and trend). The results of the test with the trend for Fisher-ADF, LLC and IPS reveal that all the variables are level stationary. The LLC unit root test with constant reveals that urbanization is level nonstationary, IPS with constant shows real gross domestic product, agricultural value-added and urbanization to be non-stationary and Fisher-ADF with constant indicates that urbanization is not stationary at level. The results of the two methods of computation for the three-unit root test suggest that most of the variables are integrated of order zero that is I (0) with the trend and constant model. However, without a trend, a few variables like agriculture and urbanization had unit root. The integration properties of the current study variables support the use of ARDL/PMG methodology for cointegration analysis. This is the premise on the merit that ARDL-PMG is flexible and robust in cases of I(0), I(1) or mixed order of series except for I(2) variables which our study has observed.

**Table 3:** Panel unit root tests.

Variables	LLC		IPS		Fisher-ADF		Integration
	constant	Trend	constant	Trend	constant	Trend	
L*CO*_*2*_	-4.05∗	-1.96∗∗	0.30	-2.19∗∗	40.10∗	43.46∗∗	I(0)
L*GDP*	-4.85∗	-18.13∗	-7.88∗	-13.14∗	39.75∗∗	277.51∗	I(0)
LAGR	-1.31∗∗	-2.18∗∗	0.01	-2.65∗	25.46	41.98∗∗	I(0)
L*URB*	-1.13	-6.35∗	1.77	-8.44∗	38.22∗∗∗	137.51∗	I(0)
L*NRT*	-3.77∗	-4.17∗	-3.40∗	-4.08∗	-3.40∗	-4.08∗	I(0)
ΔL*CO*_*2*_	-19.87∗	16.18∗	-19.89∗	-18.56∗	309.68∗	283.7∗	
ΔLG*DP*	-132.06∗	27.73∗	-47.03∗	-7.83∗	130.76∗	107.80∗	
ΔLAGR	-11.30∗	-9.33∗	-13.06∗	-11.86∗	192.17∗	160.92∗	
ΔL*URB*	-2.06∗∗	-0.59	-1.27	0.51	33.80	21.78	
ΔL*NRT*	-20.03∗	-18.40∗	-20.32∗	-19.14∗	319.63∗	292.04∗	

Notes: ∗, ∗∗ and ∗∗∗ represents are statistical significance rejection level at 1%, 5% and 10% respectively. Δ indicates first difference. Lag selection by SIC of maximum of 4 in all estimations. Here, LLC, IPS and Fisher-ADF means the Levin et al. (2002); Im et al. (2003); Fisher-ADF by Maddala & Wu (1999) panel unit root tests. Automatic lag selection is adopted for the estimations. Also, the *co*_*2*_*, gdpc, nrt, urb and ag* respectively the carbon dioxide, gross domestic product per capita, total natural rent, urbanization, agricultural value added. Here also ln represents natural logarithmic of the variables outlined.

#### 4.1.2 Panel Co-integration test

Sequel to the investigation of the stationary properties of the variables, the study deems it fit to investigate the long-run relationship between the dependent variable (carbon dioxide emissions) and the independent variables (real gross domestic product, agricultural value-added, urbanization, and total natural rent) using Pedroni and Kao co-integration tests. Out of the eight common AR coefficients (within-dimension) of the Pedroni co-integration test reported in Table 4, four coefficients indicate that the variables have a long-run relationship. Similarly, one of the three individual AR coefficients (between-dimension) confirms that there is a long-run relationship between the variables. The study further employs Kao co-integration to authenticate the result of the Pedroni co-integration test. The probability value of the Kao ADF t-statistic presented in Table 4 rejects the null hypothesis of no co-integration at 1%. This finding is in line with the submission of Appiah et al. (2018), Agboola and Bekun (2019), and Gokmenoglu and Taspinar (2018).

**Table 4:** Pedroni and Kao cointegration Results.

Alternative hypothesis: common AR coefficients (within-dimension)					
		Statistic	Prob.	W. Statistic	Prob.
Panel v-Statistic		-1.133	0.871	-1.059	0.855
Panel rho-Statistic		0.472	0.318	0.245	0.597
Panel PP-Statistic		-3.468	0.000∗∗∗	-3.126	0.000∗∗∗
Panel ADF-Statistic		-2.056	0.020∗∗	-2.023	0.022∗∗∗
Alternative hypothesis: individual AR coefficient (between-dimension)					
		Statistic	Prob.		
Group rho-Statistic		1.401	0.919		
Group PP-Statistic		-2.662	0.004∗∗∗		
Group ADF-Statistic		-0.549	0.292		

**Kao cointegration test**					
	t-Stat	Prob.			
ADF	-3.228∗∗	0.001			
Residual variance	0.043				
HAC variance	0.0287				

Note the asterisk (∗∗∗^,^∗∗ and ∗) represents statistical rejection level of null of no co-integration test statistics at 1%,5% and 10% significance level.

### 4.2 Empirical results and discussion

The PMG-ARDL technique requires variables not to be integrated of order two. Based on the results of the panel unit root tests presented in Table 3, none of the variables is stationary at the second difference. Hence, PMG-ARDL is suitable for the analysis. The long-run estimate presented in Table 5 validates the EKC hypothesis in sub-Saharan African countries. This result suggests that even though sub-Saharan Africa like many other regions of the world finds it challenging to maintain a clean environment at the early stage of economic growth possibly due to increase in greenhouse gases and other forms of carbon dioxide emission, the region performs excellently at the later stage of economic growth. Improvement in environmental quality or decline in carbon dioxide emission at the later stage of economic growth has also been obtained in other region or countries (see Agboola and Bekun, 2019; Gokmenoglu and Taspinar, 2018; Alola, Yalçiner, Alola and Saint, 2019; Gokmenoglu and Taspinar, 2018). This result may be attributed to the use of low carbon-emitting material or the availability of resources to address the problem of environmental degradation.

**Table 5:** Result of PMG-ARDL (1,1,1,1,1,1).

Model: LCO_2_ = F(LGDP, LGDP2,LAGR, LURB,LNRT)				
Variable	Coefficient	Std. Error	T-stat.	P-value
**Long run**				
LGDP	5.098∗∗∗	1.008	5.059	0.000
LGDP_2_	-0.310∗∗∗	0.068	-4.561	0.000
LAGR	-0.183∗∗	0.079	-2.331	0.020
LURB	1.579∗∗∗	0.220	7.177	0.000
LNRT	0.138∗∗	0.044	3.141	0.002
**Short run**				
ECT(-1)	-0.371∗∗∗	0.080	-4.638	0.000
ΔLGDP	-22.456	18.689	-1.202	0.230
ΔLGDP2	1.552	1.250	1.242	0.215
ΔLAGR	0.041	0.091	0.450	0.653
ΔLURB	2.415	3.526	0.685	0.494
ΔLNRT	0.023	0.053	0.436	0.663
Constant	-6.333∗∗∗	1.445	-4.382	0.000

Note the asterisk (∗∗∗^,^∗∗ and ∗) represents statistical rejection level of null of no co-integration test statistics at 1%,5% and 10% significance level. Also the fitted model is based on maximum lag 1 as suggested by Akaike information criterion With 256 observations.

The result further shows that agricultural value-added exerts a significant adverse effect on carbon dioxide emissions in the long run. In other words, a 1% increase in agricultural value-added gives rise to 0.18% decrease in carbon dioxide emission in sub-Saharan African countries. This result implies that agriculture is not only vital in the growth process of sub-Saharan African countries; it also enhances environmental quality. This result, of course, contrasts the findings of Appiah et al. (2018), Agboola and Bekun (2019), Sarkodie and Owusu (2017), as well as Gokmenoglu and Taspinar (2018) for some selected emerging economies, China, Tunisia, Nigeria, Ghana, and Pakistan respectively. The contradictory finding may be due to the difference in the method of analysis or the renewed attention giving to the environment in sub-Saharan African countries.

Urbanization and total natural resources rent have a positive and significant impact on carbon dioxide emissions in sub-Saharan African countries. This indicates that a 1% increase in urbanization and total natural rent bring about 1.58% and 0.14% increase in carbon dioxide emission in the long run respectively. An increase in the number of people in the urban areas gives rise to an increase in the use of energy resources appliances, which in turn increases carbon dioxide emissions. Similarly, the desire to boost natural resources revenue makes sub-Saharan African countries to encourage the production of energy resources, most notably, crude oil, in turn, leads to increase in the carbon emission in the region. The positive impact of urbanization is similar to the findings of Wang et al. (2019) for China but is contrary to that of Sharma (2011) and Shafiei and Salim (2014) who found a negative relationship between urbanization and emissions for 69 countries and OECD countries respectively. On the other hand, the positive impact of natural resource rent on emissions partially agrees with the findings of Bekun et al. (2019) and Balsalobre-Lorente et al. (2018) for EU-16 and EU-5 countries respectively.

In the short-run, real gross domestic product, agricultural value-added, urbanization, and total natural rent are not significant at 10% level of significance. Moreover, the lagged error correction term is significant at 1% level of significance, negative and less than one. No doubt, after every deviation of any of the independent variables, carbon dioxide emission converges to the long-run equilibrium. Not just that, the lagged error correction term authenticates the results of the panel co-integration tests, which show that a long-run relationship exists among the variables.

#### 4.2.1 Panel causality test

The direction of causality among the variables is examined using a panel heterogeneity causality test proposed by Dumitrescu and Hurlin (2012). Causality test is considered very important because it divulges the Granger causal relation and helps the policymakers to formulate policies that promote a clean environment in the sub-Saharan African countries. Bidirectional Granger causality dominates the estimated result presented in Table 6. First, there is a feedback relation between real gross domestic product and carbon dioxide emissions. So, changes in previous historical information of the real gross domestic product are capable of predicting future changes in carbon dioxide emissions. Though this result disagrees with Agboola and Bekun (2019) and Alola and Alola (2018), it is not different from the submission of Appiah et al. (2018) for some selected emerging economies.

**Table 6:** Results of the Dumitrescu and Hurlin (2012) Panel causality.

Null Hypothesis:	W-Stat.	Zbar-Stat.	Prob.
LGDP ≠>LCO_2_	7.1128∗∗∗	2.61578	0.0089
LCO_2_ ≠>LGDP	6.26784∗∗∗	1.80104	0.0717
LAGR ≠>LCO_2_	7.12573∗∗∗	2.62825	0.0086
LCO_2_ ≠>LAGR	7.06639∗∗	2.57103	0.0101
LNRT ≠>LCO_2_	5.36759	0.93298	0.3508
LCO_2_ ≠>LNRT	5.74489	1.29679	0.1947
LURB ≠>LCO_2_	9.49678∗∗∗	4.9145	9.00E-07
LCO_2_ ≠>LURB	24.106∗∗∗	19.0013	0.0000
LAGR ≠>LGDP	6.98529∗∗	2.49283	0.0127
LGDP ≠>LAGR	7.96462∗∗∗	3.43713	0.0006
LNRT ≠>LGDP	4.96563	0.5454	0.5855
LGDP ≠>LNRT	8.2139∗∗∗	3.6775	0.0002
LURB ≠>LGDP	7.05484∗∗	2.55989	0.0105
LGDP ≠>LURB	19.152∗∗∗	14.2244	0.0000
LNRT ≠>LAGR	4.8568	0.44047	0.6596
LAGR ≠>LNRT	5.03036	0.60782	0.5433
LURB ≠>LAGR	9.09908∗∗∗	4.53102	6.00E-06
LAGR ≠>LURB	10.8896∗∗∗	6.25754	4.00E-10
LURB ≠>LNRT	7.44082∗∗∗	2.93207	0.0034
LNRT ≠>LURB	9.69878∗∗∗	5.10928	3.00E-07

Note: ∗∗∗.∗∗ and ∗ means 0.01,0.05 and 0.10 statistical rejection level.

Feedback or bidirectional relationship is also observed between agricultural value-added and carbon dioxide emission. A reasonable number of existing studies (see Appiah et al., 2018; Asumadu-Sarkodie and Owusu, 2017; and Gokmenoglu and Taspinar, 2018) also report a similar result. This result implies agricultural activities such as crop and livestock farming Granger cause the level of emissions in sub-Saharan African countries. In the same way, changes in carbon dioxide emissions Granger cause changes in agriculture value-added. The study also finds evidence of a bidirectional relation between urbanization and carbon dioxide emission, which suggests that carbon dioxide emission is also caused by urbanization in sub-Saharan African countries.

Further, the study establishes a feedback relationship between agricultural value-added and real gross domestic product in sub-Saharan African countries. This reveals the importance of agrarian in the growth process of sub-Saharan African countries. There is sufficient evidence that an increase in agricultural value-added will Granger cause the growth of sub-Saharan African countries, vis-à-vis. Studies that report similar results include but not limited to Appiah et al. (2018) as well as Gokmenoglu and Taspinar (2018). Meanwhile, Agboola and Bekun (2019) submit that agricultural value-added has no Granger causal relation with carbon dioxide in Nigeria. The submission of Agboola and Bekun (2019) is, no doubt, a product of different scope and technique.

Additionally, the study uncovers the feedback relationship between urbanization and real gross domestic product, urbanization, and agricultural value-added as well as urbanization and total resources rent. Total resources rent has no Granger causal linkage with carbon dioxide emission and agricultural value. However, a unidirectional causality from real gross domestic to resources rent in sub-Saharan African countries.

## 5 Conclusion and policy implications

This study examines the role of agriculturally-induced economic performance in recovering the bluish skies of sub-Saharan African Countries. The study obtains secondary data on carbon dioxide emissions, real gross domestic product, agricultural value-added, urbanization, and total natural rent from World Bank Development Indicator for the selected panel of sub-Saharan African countries namely, Benin, Cote d'Ivoire, Mauritius, Botswana, Ethiopia, Nigeria, Cameroon, Ghana, South Africa, Congo Republic, Kenya, and Zimbabwe. The Fisher-ADF, Levin, Lin and Chu (LLC) and Im, Pesaran and Shin (IPS) are used for the stationary test, Kao and Pedroni co-integration tests for a long-run relationship, PMG-ARDL (1, 1, 1, 1, 1, 1) for impact analysis and, the Dumitrescu and Hurlin panel causality test for a causal relationship.

The study found a positive and significant relationship between gross domestic product and CO_2_ emissions over the long run. Thus, it translates that the economic output worsens the carbon emission accounting for the panel of countries especially since the protection of the environment via the use of renewable energy sources are overlooked. Interestingly, the examination asserts that agricultural value-added reduces emissions in sub-Saharan Africa while urbanization and natural resource rent both increases CO_2_ emissions in the long run. Importantly, the result of the PMG-ARDL shows that the EKC hypothesis is valid for sub-Saharan African countries. Besides, the panel causality test indicates the feedback effect is prevalent for the relationship among the variables. Most notably, the empirical result shows a bidirectional relationship between real gross domestic product and carbon dioxide emissions as well as agricultural value-added and carbon dioxide emissions in sub-Saharan Africa.

Based on the policy intuition from the study, the study suggests that sub-Saharan African countries can still use the dividend of economic growth to address the problem of environmental degradation. This will help to improve the quality of the environment thus improving the wellbeing of human and non-human aspects of the environment. Also, since empirical evidence reveals that agricultural activities avert environment hazards in the sub-Saharan African countries, thus the sub-Saharan African countries should continue to encourage the best practice of agricultural activities. As such, the region will continue to experience a significant reduction in the level of carbon dioxide emissions, thus improving environmental quality. Secondly, considering the adverse impact of natural resource rent on CO_2_ emissions, it is suggested that governments in the region pursue the exploitation of the natural resource in an environmentally efficient way to mitigate the contributions of natural resource rent to high emissions in the region. This can be achieved by regulating activities involving the exploration of natural resources in the region. The use of technology that is capable of limiting emissions from mineral exploitation will also aid in mitigating the potential harm posed to the environment.

## Declarations

### Author contribution statement

Festus Fatai Adedoyin: Contributed reagents, materials, analysis tools or data; Wrote the paper.

Andrew Adewale Alola: Conceived and designed the experiments; Performed the experiments.

Festus Victor Bekun: Analyzed and interpreted the data; Contributed reagents, materials, analysis tools or data.

### Funding statement

This research did not receive any specific grant from funding agencies in the public, commercial, or not-for-profit sectors.

### Competing interest statement

The authors declare no conflict of interest.

### Additional information

No additional information is available for this paper.
